# Comprehensive Analysis of Pertinent Genes and Pathways in Atrial Fibrillation

**DOI:** 10.1155/2021/4530180

**Published:** 2021-12-31

**Authors:** Yanzhe Wang, Wenjuan Cai, Liya Gu, Xuefeng Ji, Qiusheng Shen

**Affiliations:** Department of Cardiology, Changshu Hospital Affiliated to Nanjing University of Chinese Medicine, Changshu, 215500 Jiangsu Province, China

## Abstract

**Purpose:**

Atrial fibrillation (AF) is the most frequent arrhythmia in clinical practice. The pathogenesis of AF is not yet clear. Therefore, exploring the molecular information of AF displays much importance for AF therapy.

**Methods:**

The GSE2240 data were acquired from the Gene Expression Omnibus (GEO) database. The R limma software package was used to screen DEGs. Based on the Gene Ontology (GO), Kyoto Encyclopedia of Genes and Genomes (KEGG), and Gene Set Enrichment Analysis (GSEA) databases, we conducted the functions and pathway enrichment analyses. Then, the STRING and Cytoscape software were employed to build Protein-Protein Interaction (PPI) network and screen for hub genes. Finally, we used the Cell Counting Kit-8 (CCK-8) experiment to explore the effect of hub gene knockdown on the proliferation of AF cells.

**Result:**

906 differentially expressed genes (DEGs), including 542 significantly upregulated genes and 364 significantly downregulated genes, were screened in AF. The genes of AF were mainly enriched in vascular endothelial growth factor-activated receptor activity, alanine, regulation of histone deacetylase activity, and HCM. The PPI network constructed of significantly upregulated DEGs contained 404 nodes and 514 edges. Five hub genes, ASPM, DTL, STAT3, ANLN, and CDCA5, were identified through the PPI network. The PPI network constructed by significantly downregulated genes contained 327 nodes and 301 edges. Four hub genes, CDC42, CREB1, AR, and SP1, were identified through this PPI network. The results of CCK-8 experiments proved that knocking down the expression of CDCA5 gene could inhibit the proliferation of H9C2 cells.

**Conclusion:**

Bioinformatics analyses revealed the hub genes and key pathways of AF. These genes and pathways provide information for studying the pathogenesis, treatment, and prognosis of AF and have the potential to become biomarkers in AF treatment.

## 1. Background

Atrial fibrillation (AF) is the most frequent arrhythmia; its incidence continues to increase, reaching 10% over 75 years [1]. The frequency of atrial activation in AF is 300-600 beats/min [2]. The heartbeat frequency of AF patients is often faster and more irregular than normal people's, sometimes up to 100-160 beats/min. The prevalence of AF is also associated with other diseases, such as coronary heart disease, hypertension, and heart failure [3]. The patients with AF are mainly the elderly, and common inducing factors include rheumatic heart disease, coronary heart disease, hyperthyroidism, stroke, thromboembolism, and heart failure [4]. Stroke is one of the greatest hazards of AF. The stroke incidence in patients with nonvalvular AF is 5.6 times higher than that of average people and in patients with valvular AF is 17.6 times, and the brain caused by AF is 17.6 times. The consequences of stroke are more serious [5]. Early symptoms of AF include palpitations, fatigue, dizziness, chest discomfort, and shortness of breath [6]. AF can also cause severe morbidity and mortality. In 2017, there were 37.57 million cases of AF patients worldwide, 3.05 million new cases of AF, and 287,000 deaths. At present, medicine is still the main treatment for AF patients, which can restore sinus rhythm, reduce the ventricular rate, and prevent thromboembolic complications [7]. Nonpharmacological treatments for AF include electro conversion (conversion of sinus rhythm), radiofrequency ablation treatment, and surgical maze surgery (complete radical treatment of AF) [8].

There is no uniform classification of AF. According to its duration, it comprises paroxysmal, persistent, and permanent AF [9]. It is generally believed that paroxysmal AF refers to those who can self-convert to sinus rhythm within 7 days, generally lasting less than 48 hours. Persistent AF refers to those who last over 7 days and need drugs or an electric shock to convert to sinus rhythm. Permanent AF refers to those who cannot be converted to sinus rhythm or relapse within 24 hours after conversion. According to the presence or absence of underlying heart disease, it is divided into pathological and idiopathic AF (clinical examination without underlying heart disease). Idiopathic AF, sometimes called solitary AF, often occurs in people below 50 years old [10]. The etiology of AF is multifactorial, and its pathogenesis is not completely clarified. In recent years, many researchers have tried to find AF-related hub genes and key pathways through microarray technology. The hub genes and signaling pathways in the development of AF are still poorly understood.

Microarray data is the outcome of the gradual application of the Human Genome Project (HGP) and the rapidly developing molecular biology, leading to the development of research on the genome world, such as genomes, transcriptomes, and proteomes [11, 12]. Its advantage is that it saves laborious experiments and expensive reagents. However, the current microarray technology still has room for development. One of the emerging desires is the ability to operate and react in multiple steps. Bioinformatics is a multidisciplinary research method of biological problems, in addition to traditional biology and chemical methods usually used to solve biological problems [13]. It is to describe the technique of collecting and analyzing large amounts of biological data using computer systems. Many core technologies of bioinformatics analysis are dependent on statistics and the collection of large quantities of data usually from various experiments and labs. The applications of bioinformatics include analyses of DNA sequence, gene expression and regulation, and comparative bioinformatics of different biological genomes [14]. Through chromosome microarray analysis (CMA) DVL1, SKI, STIM1, CTNNA3, and PLN were identified as candidate genes related to the phenotype of congenital heart disease (CHD), which improved the diagnosis rate of children with CHD. Based on circRNA microarray analysis, it was found that circPDS5B and circCDC14A can be used as biomarkers to diagnose and predict the prognosis of acute ischemic stroke.

This study used bioinformatics analyses to obtain hub genes and key pathways related to AF. The microarray profile dataset GSE2240 was downloaded from the Gene Expression Omnibus (GEO) database as the research object. The finally obtained hub genes and pathways are of great significance to AF. And based on the Cell Counting Kit-8 (CCK-8) experiment, we verified the relationship between the hub gene and AF cell proliferation. This strategy is conducive to the discovery of previously neglected genes, and these findings may provide new perspectives for optimizing the treatment of AF.

## 2. Material and Methods

### 2.1. Microarray Data

Gene Expression Omnibus (GEO) (http://www.ncbi.nlm. http://nih.gov/geo) is one of the most commonly used sequencing (chip) databases in the National Center for Biotechnology Information (NCBI) (https://pubmed.ncbi.nlm.nih.gov/) [15]. And it is a public repository that can archive and freely distribute the complete set of microarrays submitted by the scientific community, next-generation sequencing, and other forms of high-throughput functional genomics data. We downloaded gene expression profile GSE2240 from the GEO database. The platform we used for GSE2240 was GPL97[HG-U133B] Affymetrix Human Genome U133B Array. The samples of GSE2240 contained 10 patients with AF and 20 people with sinus rhythm.

### 2.2. Data Processing

After downloading the gene expression profile GSE2240, we used R language software to analyze and process the database. When the genes' threshold *P* value was <0.01, they were chosen as differentially expressed genes (DEGs). At the same time, when the log_2_ (fold change) was greater than 0, the DEGs were selected as significantly upregulated genes, and when the log_2_ (FC) was less than 0, the DEGs were selected as significantly downregulated genes.

### 2.3. Gene Ontology (GO) and Kyoto Encyclopedia of Genes and Genomes (KEGG) Enrichment Analysis of DEGs

GO (http://www.geneontology.org.) is a widely used biological database, divided into three independent ontologies, namely, biological process (BP), molecular function (MF), and cellular component (CC) [16]. KEGG (http://www.genome.jp/kegg/) is used for comprehensive analysis of gene function in a knowledge base [17]. Genomic information can be linked with high-order functional information and kept in the genes database, which is a collection of gene catalogs of all fully sequenced genomes and some partial genomes with newly updated annotations. The significantly upregulated and downregulated DEGs were analyzed for GO and KEGG enrichment, respectively, through the Database for Annotation, Visualization, and Integrated Discovery (DAVID v6.8, https://david.ncifcrf.gov/tools.jsp) [18].

### 2.4. Protein-Protein Interaction (PPI) Network Analysis of DEGs

The Search Tool for the Retrieval of Interacting Genes (STRING v11.0, https://string-db.org/) database is for interaction identification between proteins on the basis of experiments, databases, text mining, and predictive bioinformatics. An interaction score of more than 0.4 was set as the standard value. Then, the Cytoscape (v3.6.0) software was used to analyze the PPI network. The genes with the highest node scores and the strongest connectivity were chosen as hub genes.

### 2.5. Gene Set Enrichment Analysis (GSEA)

GSEA uses the ranking of differential gene expression degree in two types of samples to test whether the preset gene set is enriched at the top or bottom of the ranking table and interpret biological information from another angle. The Molecular Signatures Database (MSigDB) was utilized to make Gene Set Enrichment Analysis (GSEA v3.0, http://www.broadinstitute.org/gsea/).

### 2.6. Cell Culture

We first purchased AF cells (H9C2) from American Type Culture Collection (Manassas, Virginia, USA) and then placed the cell population in DMEM medium with 10% fetal bovine serum (Gibco; Thermo Fisher Scientific, Inc.), which was then put in a humidified box containing 5% CO_2_ and maintained at 37°C for cultivation.

### 2.7. Cell Transfection

We purchased siRNA and negative control (si-NC) from Sangon (Shanghai, China), where siRNA was used to knock down the expression of the hub gene CDCA5. After that, H9C2 cells were poured into a 6-well plate and transfected with Lipofectamine 2000 (Invitrogen, California) according to the operating steps provided by the manufacturer.

### 2.8. CCK-8 Assay

In order to measure the effect of gene expression on cell proliferation, CCK-8 assay (cat. no. HY-K0301; MedChemExpress) was performed. We first added H9C2 cells to a 96-well plate at a density of 2 × 10^3^ and then poured 10 *μ*l of CCK-8 solution into each well. After a period of time, at the 24th, 48th, 72nd, and 96th hours, we used a microplate reader (BMG Labtech GmbH) to measure the optical density (OD) of the solution at 450 nm.

### 2.9. Statistical Analysis

All experiments were performed in triplicate. The results of this experiment were presented as mean ± standard deviation (SD), and SPSS 17.0 (US SPSS Inc.) was used for data analysis. It was judged statistically significant when *P* < 0.05.

## 3. Result

### 3.1. Identification of DEGs

We used R language software to analyze and process the database GSE2240. The gene expression profile GSE2240 contained myocardial samples from patients with AF (*n* = 10) and the control group with sinus rhythm (*n* = 20). We screened DEGs based on a *P* value of less than 0.01. The processing results were shown in the heat map; we obtained 906 DEGs, including 542 upregulated genes and 364 downregulated genes (Figure 1). The top 10 downregulated DEGs and top 10 upregulated DEGs are shown in Table 1.

### 3.2. GO and Pathway Enrichment Analysis of Upregulated Genes

The enrichment analysis results based on DAVID online database is shown in Figures 2 and 3. The top 10 enriched BP terms of upregulated DEGs were regulation of exit from mitosis, ganglioside metabolic process, regulation of systemic arterial blood pressure by hormone, cellular localization, natural killer cell activation, peptidyl-lysine trimethylation, glycosphingolipid catabolic process, 4-hydroxyproline metabolic process, oligosaccharide catabolic process, and interleukin-23-mediated signaling pathway (Figure 2(a)). For CC, the upregulated DEGs were mainly enriched in GO terms of clathrin coat, perinuclear endoplasmic reticulum, microtubule minus-end, mitotic spindle, ionotropic glutamate receptor complex, mitotic spindle pole, INO80-type complex, microtubule end, dendrite membrane, and GABA-A receptor complex (Figure 2(b)). For MF, the upregulated DEGs in AF were chiefly distributed in GO terms of diacylglycerol kinase activity, rac guanyl-nucleotide exchange factor activity, phosphatidylinositol phosphate phosphatase activity, hydroxymethyl-, formyl- and related transferase activity, alpha-N-acetylneuraminate alpha-2,8-sialyltransferase activity, SH3 domain binding, aldehyde-lyase activity, phosphatidylinositol phosphate 4-phosphatase activity, and vascular endothelial growth factor-activated receptor activity (Figure 2(c)). The most significantly enriched pathways of upregulated DEGs analyzed by KEGG analysis were the HIF-1 signaling pathway, one carbon pool by folate, alanine, aspartate and glutamate metabolism, nicotine addiction, phenylalanine, tyrosine, and tryptophan biosynthesis, glyoxylate and dicarboxylate metabolism, synaptic vesicle cycle, amyotrophic lateral sclerosis (ALS), vibrio cholerae infection, and phosphatidylinositol signaling system (Figure 2(d)).

### 3.3. GO and Pathway Enrichment Analysis of Downregulated Genes

GO and KEGG analyses are considered to be powerful tools for revealing the biological mechanisms or functional pathways of genomics or transcriptional observation patterns. The top 10 enriched BP terms of downregulated DEGs were modification-dependent protein catabolic process, protein localization to the nonmotile cilium, muscle cell differentiation, positive regulation of deacetylase activity and endothelial cell migration, iron ion transport, regulation of synapse assembly, regulation of histone deacetylase activity, protein monoubiquitination, and skeletal muscle tissue development (Figure 3(a)). For CC, the downregulated DEGs were chiefly enriched in GO terms of nuclear heterochromatin, nuclear speck, endoplasmic reticulum quality control compartment, heterochromatin, Cul3-RING ubiquitin ligase complex, euchromatin, vacuole, spindle midzone, focal adhesion, and nuclear body (Figure 3(b)). For MF, the downregulated DEGs were chiefly enriched in GO terms of iron ion transmembrane transporter activity, ubiquitin-protein ligase activity, ubiquitin-protein transferase activity, methylation-dependent protein binding, oxalate transmembrane transporter activity, ubiquitin-like protein ligase activity, transcription regulatory region DNA binding, sulfate transmembrane transporter activity, methylated histone binding, and 3′,5′-cyclic-GMP phosphodiesterase activity (Figure 3(c)). The most marked pathways of downregulated DEGs analyzed by KEGG analysis were mineral absorption, nonalcoholic fatty liver disease (NAFLD), AMPK signaling pathway, tight junction, hypertrophic cardiomyopathy (HCM), T cell receptor signaling pathway, circadian rhythm, vitamin B6 metabolism, spliceosome, and GnRH signaling pathway (Figure 3(d)).

### 3.4. Signaling Pathways of Genes Associated with MF

We further carried out GSEA on the database GSE2240. It was observed that these genes from 10 patients with AF were positively correlated with aldosterone-regulated sodium reabsorption (Figure 4(a)), olfactory transduction (Figure 4(b)), and arginine and vibrio cholerae infection (Figure 4(c)) signaling pathways compared to the genes from a person with sinus rhythm.

### 3.5. PPI Network Analysis of Upregulated Genes

We used the selected upregulated DEGs to build a PPI network, and Cytoscape software was used for analyzing the PPI network. 404 nodes and 514 protein pairs were acquired with a combined score of >0.4 based on the STRING database (Figure 5). The higher the degree was, the more closely the gene was associated with AF. ASPM (degree = 19), DTL (degree = 17), STAT3 (degree = 17), ANLN (degree = 16), and CDCA5 (degree = 16) were identified as key upregulated genes. Furthermore, as shown in the box plot diagram, the expression levels of ASPM, DTL, STAT3, ANLN, and CDCA5 in myocardial tissue of AF were significantly higher than those in myocardial tissue of sinus rhythm (Figures 6(a)–6(e)). We could summarize that ASPM, DTL, STAT3, ANLN, and CDCA5 were upregulated hub genes of AF.

### 3.6. PPI Network Analysis of Downregulated Genes

Also, we used the selected downregulated DEGs to construct a PPI network, and the Cytoscape software was used to analyze the PPI network. 327 nodes and 301 protein pairs were acquired with a combined score of >0.4 through the STRING database (Figure 7). CDC42 (degree = 23), CREB1 (degree = 16), AR (degree = 13), and SP1 (degree = 10) were identified as key downregulated genes. As shown in the box plot diagram, the expression levels of CDC42, CREB1, AR, and SP1 in myocardial tissues of AF were significantly lower than those in myocardial tissues of sinus rhythm (Figures 8(a)–8(d)). We could summarize that CDC42, CREB1, AR, and SP1 were downregulated hub genes of AF.

### 3.7. CDCA5 Knockdown Prevented Cell Proliferation

On the basis of exploring the effects of the hub genes on the proliferation of H9C2, we knocked down the expression of the hub gene through siRNA. As shown in Figure 9(a), CDCA5 gene knockdown prevented H9C2 proliferation compared to the negative control (si-NC).

## 4. Discussion

AF accounts for about one-third hospitalizations for arrhythmia and is the most common arrhythmia [19]. Many researchers believe that inflammation, neurohormonal disorders, and cardiovascular diseases, such as valvular diabetes, hypertension, congestive heart failure, myocardial infarction, and genetic factors, are “regulators” that can induce AF [20, 21]. Among them, genetic factors have key functions in AF oncogenesis. The heritability of polygenic debt for AF is estimated to be 0.62. The focus of bioinformatics research is mainly reflected in two aspects: genomics and proteomics [22]. It is the science of maintaining, retrieving, and delving biological information using computers as tools in the research of life sciences. According to the role of biomolecules in gene regulation, the internal laws of diagnosis and treatment of human diseases are described [23]. Its research goal is to reveal the “complexity of genome information structure and the fundamental laws of genetic language” and explain the genetic language of life. Bioinformatics has become an important part of the development of the entire life sciences and has become the forefront of life science research [24].

Based on the GSE2240 database, a total of 906 DEGs related to the AF process were identified. In order to further analyze the potential mechanisms involved in DEGs, we conducted a functional and pathway enrichment analysis. Our research results found that vascular endothelial growth factor-activated receptor activity and alanine were the significantly enriched pathways of upregulated DEGs. Mezache et al. pointed out that the effect of vascular endothelial growth factor on the heart was multifactorial. Inflammation, vascular leakage, and related tissue edema are common sequelae of AF [25]. Alanine constitutes the basic unit of protein and is one of the 20 amino acids that make up human protein. The role of alanine is to produce sugar from dietary protein. For downregulated DEGs, regulation of histone deacetylase activity and hypertrophic cardiomyopathy (HCM) were the significant enriched pathways. Studies by Evans and others have shown that histone deacetylase activity was significantly upregulated in the heart remodeling model, which had the risk of heart diseases, such as AF, myocardial infarction, and myocardial failure [26]. Xu et al. found that AF was the most frequent persistent arrhythmia in patients with HCM. HCM patients with AF have upregulated morbidity and mortality because of heart failure and stroke. HCM patients are more prone to develop AF, and the existence of AF is associated with an increase in morbidity and mortality [27]. In summary, DEGs may affect the activity of receptors activated by vascular endothelial growth factor, the synthesis of alanine, and the regulation of histone deacetylase activity, which ultimately leads to the progression of AF.

Through PPI network analysis, we found that the genes most associated with AF were ASPM, DTL, STAT3, ANLN, CDCA5, CDC42, CREB1, AR, and SP1. The full name of ASPM is the assembly factor for spindle microtubules. ASPM-related diseases include microcephaly 5 and primary autosomal recessive microcephaly [28]. GO annotations related to this gene include binding and calmodulin binding. EHBP1 is a crucial paralog of this gene. Szczepanek et al. studied that STAT3 was initially identified as an IL-6-induced acute-phase gene transcription activator. The normal cardiac function requires the expression of STAT3. The expression of STAT3 transcription factor in the heart has a cardioprotective effect and reduces reactive oxygen species [29]. SP1 is a protein-coding gene that is linked with Huntington's disease and embryonal carcinoma [30]. Toll-like receptor signaling pathways and G-beta gamma signaling are its pertinent pathways. GO annotations include DNA-binding transcription factor activity and sequence-specific DNA binding. The mechanism of action of the hub gene and the correlation between its expression level and the clinical parameters of AF need to be further studied.

## 5. Conclusion

This study uses systematic bioinformatics analyses to obtain the pivotal genes and key pathways related to AF. As a research object, the microarray profile data GSE2240 is acquired in the GEO database. A total of 542 upregulated DEGs and 364 downregulated DEGs were identified. GO, KEGG, and GSEA analyses were used to analyze the potential functions of DEGs. Hub genes were identified based on the PPI network, including ASPM, DTL, STAT3, ANLN, CDCA5, CDC42, CREB1, AR, and SP1. These pivotal genes and key pathways are helpful to the AF research progress and can be used as AF potential diagnosis biomarkers, treatment, and prognosis. Not only that, we also find that knocking down the expression of CDCA5 inhibits the proliferation of AF cells (H9C2). These findings will benefit the development of AF diagnosis and treatment.

## Figures and Tables

**Figure 1:** Hierarchical clustering heat map of all DEGs in AF. Yellow is upregulated DEGs, and purple is downregulated DEGs.

**Figure 2:** GO and KEGG enrichment analysis of upregulated DEGs in AF. (a–c) Top 10 BP, CC, and MF terms in which the upregulated DEGs were enriched. (d) Top 10 KEGG pathways in which the upregulated DEGs were enriched.

**Figure 3:** GO and KEGG enrichment of downregulated DEGs in AF. (a–c) Top 10 BP, CC, and MF terms in which the upregulated DEGs were enriched. (d) Top 10 KEGG pathways in which the downregulated DEGs were enriched.

**Figure 4:** GSEA analysis of pathways related with AF based on dataset GSE2240. (a) The gene set of aldosterone-regulated sodium reabsorption was significantly enriched in AF patient samples. (b) The gene set of olfactory transduction was significantly enriched in AF patient samples. (c) The gene set of vibrio cholerae infection was significantly enriched in AF patient samples.

**Figure 5:** The constructed PPI network for upregulated DEGs. The PPI network contains 404 nodes and 514 edges. Nodes mean proteins and edges mean the interaction of proteins.

**Figure 6:** The expression level of (a) STAT3, (b) ASPM, (c) ANLN, (d) CDCA5, and (e) DTL in myocardial tissues of AF was significantly higher than that in myocardial tissues of sinus rhythm.

**Figure 7:** The constructed PPI network for downregulated DEGs. The PPI network contains 327 nodes and 301 edges. Nodes mean proteins and edges mean the interaction of proteins.

**Figure 8:** The expression levels of (a) SP1, (b) AR, (c) CDC42, and (d) CREB1 in myocardial tissues of AF were significantly lower than those in myocardial tissues of sinus rhythm.

**Figure 9:** CDCA5 knockdown inhibited the proliferation of H9C2 cells. The *x*-axis is the number of days, and the *y*-axis is the OD value at 450 nm corresponding to the number of days. ^∗^*P* < 0.05.

**Table 1:** Log-fold changes of the top10 upregulated DEGs and top10 downregulated DEGs in the sinus rhythm control group and atrial fibrillation patient samples.

Gene symbol	Gene title	log_2_ FC	*P*	Expression
SEL1L3	SEL1L family member 3	0.060340007	2.25*E* − 07	Upregulated
DHRS9	Dehydrogenase/reductase 9	0.188569525	7.01*E* − 07	Upregulated
FLT4	Fms-related tyrosine kinase 4	0.099135639	7.40*E* − 07	Upregulated
BICD1	BICD cargo adaptor 1	0.163528177	7.89*E* − 07	Upregulated
LINC00608	Long intergenic non-protein-coding RNA 608	0.043723792	1.29*E* − 06	Upregulated
RNF216	Ring finger protein 216	0.074128631	1.82*E* − 06	Upregulated
DHRS13	Dehydrogenase/reductase 13	0.045246216	2.16*E* − 06	Upregulated
PRR11	Proline-rich 11	0.056029931	3.58*E* − 06	Upregulated
MAD2L2	MAD2 mitotic arrest deficient-like 2 (yeast)	0.040471973	4.38*E* − 06	Upregulated
ATP1B4	ATPase Na+/K+ transporting family member beta 4	0.307563341	4.45*E* − 06	Upregulated
GALNT16	Polypeptide N-acetylgalactosaminyltransferase 16	-0.098686876	2.84*E* − 08	Downregulated
HCN4	Hyperpolarization-activated cyclic nucleotide-gated potassium channel 4	-0.082582678	1.51*E* − 07	Downregulated
MASP1	Mannan-binding lectin serine peptidase 1	-0.102728211	2.31*E* − 06	Downregulated
LGR6	Leucine-rich repeat-containing G protein-coupled receptor 6	-0.103112526	3.33*E* − 06	Downregulated
LOC102725271///NTM	Neurotrimin-like///neurotrimin	-0.202137537	5.13*E* − 06	Downregulated
CLSTN2	Calsyntenin 2	-0.131561085	6.84*E* − 06	Downregulated
TMEM245	Transmembrane protein 245	-0.089869756	8.86*E* − 06	Downregulated
BTBD7	BTB domain-containing 7	-0.073546467	9.78*E* − 06	Downregulated
ZNF521	Zinc finger protein 521	-0.095026053	1.25*E* − 05	Downregulated
FNDC5	Fibronectin type III domain-containing 5	-0.076766249	1.62*E* − 05	Downregulated

## Data Availability

The datasets used and/or analyzed during the current study are available from the corresponding author on reasonable request.

## References

[1] Moss H. M. (2009). *Knowledge of Coumadin Use and Vitamin K Interaction in Atrial Fibrillation Patients*.

[2] Chatap G., Giraud K., Vincent J. P. (2002). Atrial fibrillation in the elderly. *Drugs & Aging*.

[3] Friesen A. D. (2007). Treatment of atrial fibrillation. *Heart*.

[4] Asadpour P. M., Pardal A. H., Afshar M., Beyranvand M. R. (2010). Comparing the serum level of apelin in patients with lone atrial fibrillation and their control group. *Pajoohandeh Journal*.

[5] Hart R. G., Sherman D. G., Easton J. D., Cairns J. A. (1998). Prevention of stroke in patients with nonvalvular atrial fibrillation. *Neurology*.

[6] Namazee M. H., Rohani-Sarvestani H. R., Serati A. R. (2008). The early presentation of atrial myxoma with acute myocardial infarction. *Archives of Iranian Medicine*.

[7] Zhang C. T., Lei R., Geriatrics D. O. (2017). Treatment for atrial fibrillation in the elderly. *Chinese Journal of Practical Internal Medicine*.

[8] Gomes M. J., Pagan L. U., Okoshi M. P. (2019). Non-pharmacological treatment of cardiovascular disease|importance of physical exercise. *Arquivos Brasileiros de Cardiologia*.

[9] Kamath S., Chin B., Blann A. D., Lip G. (2002). A study of platelet activation in paroxysmal, persistent and permanent atrial fibrillation. *Blood Coagulation & Fibrinolysis*.

[10] Chimenti C., Russo M. A., Carpi A., Frustaci A. (2010). Histological substrate of human atrial fibrillation. *Biomedicine & Pharmacotherapy*.

[11] Burke H. B. (2000). Discovering patterns in microarray data. *Molecular Diagnosis*.

[12] Jane H. C. (2004). Integrated transcriptome and proteome data: the challenges ahead. *Briefings in Functional Genomics & Proteomics*.

[13] van Driel M. A., Brunner H. G. (2006). Bioinformatics methods for identifying candidate disease genes. *Human Genomics*.

[14] Kasabov N. Bioinformatics: a knowledge engineering approach.

[15] Barrett T., Wilhite S. E., Ledoux P. (2011). NCBI GEO: archive for functional genomics data sets–update. *Nucleic Acids Research*.

[16] Blake J. A., Chan J., Kishore R., Sternberg P. W., Li Y. (2015). Gene Ontology Consortium: going forward. *Nucleic Acids Research.*.

[17] du J., Yuan Z., Ma S., Song J., Xie X., Chen Y. (2014). KEGG-PATH: Kyoto encyclopedia of genes and genomes-based pathway analysis using a path analysis model. *Molecular Biosystems Electronic Edition*.

[18] Francesco T., Kristen P. G., John B., John S. C., Christian M. (2015). *Pathways Identified by the Database for Annotation, Visualization and Integrated Discovery (DAVID Version 6.7)*.

[19] Lugero C., Kibirige D., Kayima J., Mondo C. K., Juergen F. (2016). Atrial fibrillation among the black population in a Ugandan tertiary hospital.. *International Journal of General Medicine*.

[20] Kato K., Oguri M., Hibino T. (2007). Genetic factors for lone atrial fibrillation. *International Journal of Molecular Medicine*.

[21] Andrew M., Nelson B. P. (2006). Atrial fibrillation. *Mount Sinai Journal of Medicine*.

[22] Al-Haggar M. M., Khair-Allaha B. A., Islam M. M., Mohamed A. S. (2013). Bioinformatics in high throughput sequencing: application in evolving genetic diseases. *Journal of Data Mining in Genomics & Proteomics.*.

[23] Alberti S., Hyman A. A. (2021). Biomolecular condensates at the nexus of cellular stress, protein aggregation disease and ageing. *Nature Reviews. Molecular Cell Biology*.

[24] Rao V. S., Das S. K., Rao V. J., Srinubabu G. (2008). Recent developments in life sciences research: role of bioinformatics. *African Journal of Biotechnology*.

[25] Mezache L., Struckman H. L., Greer-Short A. (2020). Vascular endothelial growth factor promotes atrial arrhythmias by inducing acute intercalated disk remodeling. *Scientific Reports*.

[26] Evans L. W., Bender A., Burnett L. (2020). Emodin and emodin-rich rhubarb inhibits histone deacetylase (HDAC) activity and cardiac myocyte hypertrophy. *The Journal of Nutritional Biochemistry*.

[27] Xu H., Wang J., Yuan J. (2020). Implication of apnea-hypopnea index, a measure of obstructive sleep apnea severity, for atrial fibrillation in patients with hypertrophic cardiomyopathy. *Journal of the American Heart Association*.

[28] Gul A., Hassan M. J., Mahmood S. (2006). Genetic studies of autosomal recessive primary microcephaly in 33 Pakistani families: novel sequence variants in ASPM gene. *Neurogenetics*.

[29] Szczepanek K., Chen Q., Derecka M. (2011). Mitochondrial-targeted signal transducer and activator of transcription 3 (STAT3) protects against ischemia-induced changes in the electron transport chain and the generation of reactive oxygen species. *Journal of Biological Chemistry*.

[30] Chen-Plotkin A. S., Sadri-Vakili G., Yohrling G. J. (2006). Decreased association of the transcription factor Sp1 with genes downregulated in Huntington’s disease. *Neurobiology of Disease*.

